The article "“Green” Synthesis of Metallic Nanoparticles by Sonoelectrochemical and Sonogalvanic Replacement Methods" was published in 2021. Journal: Bioinorg Chem Appl.

# “Green” Synthesis of Metallic Nanoparticles by Sonoelectrochemical and Sonogalvanic Replacement Methods

**DOI:** 10.1155/2021/9830644

**Published:** 2021-11-28

**Authors:** Оrest Kuntyi, Galyna Zozulya, Andriy Kytsya

**Affiliations:** ^1^Department of Chemistry and Technology of Inorganic Substances, Lviv Polytechnic National University, Bandery Str. 12, Lviv 79013, Ukraine; ^2^Department of Physical Chemistry of Fossil Fuels of the Institute of Physical-Organic Chemistry and Coal Chemistry Named After L. M. Lytvynenko of the National Academy of Sciences of Ukraine, Naukova Str. 3а, Lviv 79060, Ukraine

## Abstract

The main features of the “green” synthesis of metallic nanoparticles (MNPs) by the sonoelectrochemical methods are manufacturability, environmental friendliness, and the possibility of controlling the geometry of the forming particles. The electrochemical reduction technique allows efficiently designing the metal nanoparticles and provides the control of the content of components of bimetallic nanoparticles, as well as minimizing the number of precursors in working solutions. Due to the generation of turbulence, microjets, and shock waves, ultrasound increases mass transfer and formation of radicals in aqueous solutions and, accordingly, accelerates the processes of nucleation and growth of MNPs. Therefore, this hybrid method, which combines electrolysis and ultrasound, has attracted the interest of researchers in the last two decades as one of the most promising techniques. The present work presents a short analysis of the reference literature on sonoelectrochemical synthesis of metallic and bimetallic nanoparticles. The main factors influencing the geometry of nanoparticles and their size distribution are analyzed. The use of pulsed ultrasound and pulsed current supply during sonoelectrochemical synthesis is especially effective in designing MNPs. Emphasis is placed on the role of surfactants in the formation of MNPs and sacrificial anodes in providing the algorithm: “anodic dissolution-electrochemical reduction of metal-nucleation and formation of МNPs.” It is noted that ultrasound allows synthesizing the MNPs and M_1_M_2_NPs during the galvanic replacement, and an analogy of the formation of nanoparticles by sonogalvanic replacement and sonoelectrochemical method is shown.

## 1. Introduction

Metal nanoparticles are widely used in biomedicine [1–5], biosensors [4, 6, 7], catalysis [1, 8], and other fields. The nanoparticles of noble metals are the most studied in terms of the synthesis methods, as well as physicochemical and functional properties. AgNPs have a special place among all noble metals because they are characterized by high antimicrobial and anti-inflammatory activity and antitumor action. This gives the possibility of effectively applying them in the pharmaceutical and cosmetic industry; antibacterial, antiviral, and cancer therapy; tissue engineering; and other areas of biomedicine (Figure 1). Using the AuNPs [3] and PtNCs [4] for the treatment of cancer and bacterial diseases gave encouraging results in the last decade. In addition, AuNPs and PtNCs are considered as a new effective class of chemotherapeutics in the treatment of hematopoietic, lung, and hepatocellular malignant tumors.

Nanoparticles and nanoclusters of noble metals are effective in detecting the biological agents and therefore play a very important role in biomedicine. Thus, in [6], the advantages of plasmonic AgNPs, AuNPs, and PtNPs for the colorimetric sensing applications in drugs assays in pharmaceutical and biological samples are described. The use of gold nanoparticles in the chemiluminescence technique showed a high sensitivity for the detection of biological agents [7].

Functional properties of MNPs, especially their biological activity, depend on both the nature of the metal and the geometry of the particles, that is, shape (sphere, rod, nanoshell, nanostar, etc.) and size (from 1 to 100–150 nm) [1–7]. The geometry of MNPs determines their excellent biocompatibility and optical (caused by the surface plasmon resonance phenomenon) and catalytic properties (Figure 2). The different nanoeffects of the size and shape of metal nanoparticles mentioned above give the possibility of effectively using the MNPs in the biosensors.

Taking into account the requirement in such materials, as well as the dependence of their functional properties on the geometry of the particles and their composition, the choice of the correct method of MNPs' synthesis is very important. After all, in the triad, *the method of synthesis* *⟶* *geometry MNPs (and composition for M*_*1*_*M*_*2*_*NPs)* *⟶* *functional properties*, the first component is decisive. The processes of obtaining of MNPs and M_1_M_2_NPs should correspond to the following basic modern criteria: (1) the control of the geometry and the composition (for binary) of nanoparticles; (2) “green” synthesis; and (3) manufacturability. Regardless of the method of synthesis (chemical [9, 10], electrochemical [11, 12], or physicochemical [13]), the controlled synthesis is the main condition for its effectiveness. “Green” synthesis is based on the use of nontoxic precursors, primarily reducing agents and surfactants of natural origin, such as plant extracts [9] and microorganisms [10]. “Green” synthesis also includes the electrochemical methods due to the cathodic reduction of metal ions and the use of nontoxic surfactants [11–13].

Manufacturability of synthesis of MNPs and M_1_M_2_NPs means, first of all, the maintenance of a high rate of processes. This is provided by electrochemical microplasma [13] and ultrasound [14–21]. Herein, we will consider ultrasound as one of the effective factors of MNPs engineering intensification.

In the last two decades, the interest in the use of ultrasound in nanomaterials preparation is greatly increased [14–21]. This is primarily caused by the complex effects of the ultrasonic field in aqueous solutions [22] such as (1) generation of turbulence, microjets, and shock waves; (2) increased mass transfer; and (3) formation of radicals in aqueous solutions. These effects have been successfully used in sonoelectrochemical deposition of nanostructured metal coatings [21, 23–28], preparation of composites [21, 29], sonoelectrochemical synthesis of colloidal solutions of metal nanoparticles [15, 17, 20], and so on. The specificity of the synthesis of colloidal solutions of metal nanoparticles is due to the multifactorial and mutual influence of ultrasound and electrolysis on the formation of MNCs and MNPs in solutions [17, 19]. Such complex impact of ultrasound and electrolysis makes it possible to provide a high rate of controlled synthesis of nanoparticles of metals of different nature (Table 1). Additionally, it should be noted that such technique is applicable for the synthesis of the metals characterized by positive values of the standard electrode potential (copper [30–33], noble metals [34–53]) and the metals characterized by negative values of *E*^0^ (iron [54, 55], nickel [56], tungsten [57], magnesium [58], aluminum [59]).

Also, sonoelectrochemical techniques are effective in obtaining the bimetallic nanoparticles (M_1_M_2_NPs) and provide the controlled composition of binary systems. For example, such a method can be used for the synthesis of M_1_M_2_NPs containing the components characterized by close values of standard electrode potentials (Fe, Co, Ni [56, 60–62]) as well as nanosystems which significantly are differed in the values of *E*^0^ (Fe and Cr [63], Cu and Ni [64], Cu and Pt [65], Pd and Fe [66], Au and Ag [66]). Moreover, applying this technique, it is possible to control the size of nanoparticles during the synthesis (Table 2).

In nanomaterial science, galvanic replacement is used for obtaining the metal nanostructures on the surface of the sacrificial substrate [69–73] and submicron metal powders [74]. Sacrificial nanoscale metal is required for the synthesis of MNPs [75]. In [76–79], MNPs were synthesized using the sacrificial metal in the form of sheets, plates, or foils via the combining method of galvanic replacement and ultrasound in solutions containing the surfactants. Ultrasound is effective in the synthesis of M_1_M_2_NPs by galvanic replacement [80–86], and the sizes of obtained nanoparticles are in the range from a few nanometers up to 100 nm (Table 3). Sonogalvanic replacement also can be attributed to the sonoelectrochemical technique because the GR process proceeds via an electrochemical mechanism [69–72]. On the surface of the sacrificial metal, there are anode and cathode areas, where the electrons are “generated” due to electrochemical dissolution with the subsequent reduction of the metal ions and the MNPs formation. Therefore, the effect of the ultrasonic field on the electrochemical processes during galvanic replacement is similar to its effect during electrolysis.

An effect of “cavitation” is the main factor of ultrasound influencing the processes which occur (1) in the bulk of the electrolyte, (2) in the double electric layer, and (3) on the surface of the electrodes. All of these processes take place during the sonoelectrochemical synthesis of MNPs. The main factors contributing to the effective synthesis of MNPs are the following:

(1). The destruction of cavitation bubbles causes high local temperatures and pressures. As a result, water is sonolized [14] and the radicals H^∗^ and ^∗^OH (equation (1)) as well as the products of their interaction (equation (2)) are formed. In the presence of surfactants in the solution (which are commonly used as stabilizers of MNCs and MNPs), organic radicals R· (equation (3)) are also formed. Such radicals and products reduce the metal ions (equations (4)–(6)), primarily noble metals, which are characterized by high values of standard electrode potentials. Atoms M^0^ combine into nanoclusters and nanoparticles (equation (7)). Thus, a typical sonochemical synthesis of MNPs takes place in the bulk of electrolyte:
  (1) $$\begin{array}{c} {\text{H}}_{2}\text{O}⟶\text{H}+\text{OH} \end{array}$$
  (2) $$\begin{array}{c} \text{HO}+\text{OH}⟶{\text{H}}_{2}{\text{O}}_{2} \end{array}$$
  (3) $$\begin{array}{c} \text{RH}+\text{OH}\left(\text{H}\right)⟶\text{R}+{\text{H}}_{2}\text{O}\left({\text{H}}_{2}\right) \end{array}$$
  (4) $$\begin{array}{c} {\text{M}}^{\text{n}+}+\text{nH}⟶{\text{M}}^{0}+{\text{nH}}^{+} \end{array}$$
  (5) $$\begin{array}{c} {\text{M}}^{\text{n}+}+\text{nR}⟶{\text{M}}^{0}+{\text{nR}}^{\prime }+{\text{nH}}^{+} \end{array}$$
  (6) $$\begin{array}{c} {\text{M}}^{\text{n}+}+{\text{nH}}_{2}{\text{O}}_{2}⟶M^{0}+{\text{nH}}_{2}O+\frac{\text{n}}{2}*{\text{O}}_{2} \end{array}$$
  (7) $$\begin{array}{c} {\text{mM}}^{0}⟶{\text{M}}_{\text{m}}\left(\text{MNCs}\right)⟶\cdots ⟶\text{MNPs} \end{array}$$
(2) In the ultrasound field, a thinning of the electrode diffusion layer thickness occurs. It causes a great enhancement in mass transport near the electrode, thereby accelerating the rate of the electrochemical reactions. At the same time, the values of currents of anodic dissolution of sacrificial metal [41, 42, 45, 49, 54] and cathode currents of metal ion reduction [41] increase significantly. Such a phenomenon leads to the increase in the rate of nucleation and, respectively, the formation of the smaller particles in comparison with the synthesis without US (Figure 3).
(3) The most described sonoelectrochemical synthesis of MNPs combines the pulsed electrolysis and pulsed ultrasound accordingly with the following algorithm [33, 34, 36]: *1. Time of electrolysis (τ*_*on*_) *⟶* *2. Time of ultrasound (τ*_*US*_) *⟶* *3. Pause of electrolysis and ultrasound (τ*_*off*_) (Figure 4).

Ultrasound periodically performs the function of “shaking” of MNPs from the cathode surface after their deposition during the current pulse. Moreover, the ultrasonic horn is periodically used as the vibrating working electrode, that is, as “sonoelectrode” in a three-electrode setup [17, 34]. During the pause of electrolysis *(τ*_off_), in addition to the “shaking” of MNPs, the diffusion of metal ions to the cathode occurs (Figure 5). It was noted that the time of the ultrasound (*τ*_US_) is a period of peculiar ablation of metallic nuclei from the cathodic surface [53].

Sonoelectrochemical synthesis of metallic nanoparticles as a hybrid technique significantly predominates the sonochemical and electrochemical methods in terms of the rate of the process. In addition, it is controllable and allows obtaining mono- and bimetallic nanoparticles of a wide range of sizes from 2 to 100 nm (Tables 1 and 2). However, the techniques described in the references differ in the constructions of sonoelectrochemical cells, power, and frequency of ultrasound applied and the constructions of current supply and modes of electrolysis. Therefore, the purpose of this review is to offer a systematic analysis of the references on sonoelectrochemical synthesis of metallic nanoparticles over the past two decades and provide the guidelines of operating conditions to maximize the beneficial effects.

## 2. Sonoelectrochemical Synthesis of Metallic Nanoparticles

The vast majority of reported methods of sonoelectrochemical synthesis of MNPs and M_1_M_2_NPs are based on the use of corresponding simple or complex salts as the precursors of metal ions (Tables 1 and 2). Only in some references, the source of metal ions is sacrificial anodes; for example, silver electrodes were applied in solutions of HCl [38] and NaPA [41] for the synthesis of AgNPs. Most of the sonoelectrochemical syntheses of metallic nanoparticles are based on the use of surfactants to stabilize of MNPs and M_1_M_2_NPs. Usually the polymeric substances containing different functional groups are used as the surfactants, for example, PVP [32, 33, 37, 39, 43, 52], PVA [31], NaPA [41, 62], and rhamnolipid [42]. In some cases, the role of the surfactant can play the molecules of the solvent, for example, THF [54, 58, 59].

### 2.1. Sonoelectrochemical Synthesis of MNPs

MNPs of the wide range of the standard electrode potentials values (Table 1) can be obtained using the sonoelectrochemical technique. In the presence of surfactants in solutions, metal ions of simple salts exist in the form of complexes. Thus, in PVP solutions, Cu(II) [33] or Ag (I) ions form complexes due to electron-donor atoms of the oxygen and nitrogen of the pyrrolidone fragment of the polymer molecule of PVP, which leads to the formation of a bond via the donor-acceptor mechanism: O: *⟶* □Ag(+) and (or) N: *⟶* □Ag(+). Therefore, in PVP solution, the complexes of Ag(І) localized in the polymer chain with a bidentate ligand are formed (Figure 6(a)). Complexes formed in NaPA solutions are presented in Figure 6(b).

#### 2.1.1. CuNPs

The main difficulty of sonoelectrochemical synthesis of CuNPs is the tendency for easy oxidation of copper in aqueous solutions. Even an inert atmosphere does not prevent the formation of CuO because, in aqueous solutions hydroxyl radicals (equation (1)), H_2_O_2_ (equation (2)) and O_2_ (equation (6)) are formed due to sonolysis and oxidize CuNPs. Therefore surfactants (PVP [30, 32, 33] or PVA [31]) are used as a capping agent. In addition, еlectron-donor atoms of the oxygen and nitrogen of the pyrrolidone fragment of the polymer molecule of PVP form bonds with Cu^2+^ ions via donor-acceptor mechanism: O: *⟶* Cu^2+^ and (or) N: *⟶* Cu^2+^ [33]. Therefore, PVP-Cu^2+^ complexes are formed, which are transformed into an intermediate neutral PVP−Cu^0^ complex, and the surface PVP−CuNPs complex is formed after the cathodic reduction of Cu^2+^ to Cu^0^. Synthesis of CuNPs is performed by well-known pulsed sonoelectrochemical method in accordance with the following protocol: *electrolysis (τ*_*on*_) *⟶* *ultrasound (τ*_*US*_) *⟶* *рause of electrolysis and ultrasound (τ*_*off*_). The size of nanoparticles depends on the following main factors: sonication power, current density, temperature, experiment duration. In [30], an optimal range of values for the sonication power was shown. Thus, at 20 W, complete separation of precipitate from the sonoelectrode is not provided, but ultrasonic power more than 90 W causes a significant increase in the size of CuNPs. Such phenomenon is due to overheating of the solution, but the increase in temperature is undesirable for obtaining small nanoparticles. For example, at sonoelectrochemical synthesis at 15°С, CuNPs with an average size of 17 nm are formed, while at 50°С, the size of particles is increased to 62 nm [33]. Therefore, ultrasonic power should be sufficient to ensure complete removal of nanoparticle sediment from the sonoelectrode but should not be too high to cause the overheating of solution. The influence of current density is also significant. A decrease in the size of CuNPs with decreasing the value of i_сathode_ was noted; for example, the mean diameter of CuNPs reduced from ∼800 nm to ∼45 nm with decreasing i_сathode_ from 760 mA·cm^−2^ to 240 mA·cm^−2^ [30]. The tendency to decrease the size of nanoparticles with increasing i_сathode_ is also shown by [33]: at 55, 70, and 100 mA·cm^−2^, CuNPs with mean diameters of 29, 24, and 10 nm, respectively, were obtained.

#### 2.1.2. AgNPs

Sonoelectrochemical synthesis of AgNPs is carried out mainly in solutions containing surfactants. Most of reported surfactants are ligands, so the reduction from complexes such as Ag(І)−NTA [34, 36], Ag(І)−EDTA [35], Ag(І)−PVP [37, 39], Ag(І)−РА^−^ [41] to Ag(0) occurs. In the formation of nanoclusters and nanoparticles, the surfactants participate in the formation of surface complexes and, accordingly, play the role of AgNPs stabilizers. The following three variants of sonoelectrochemical synthesis of AgNPs are described in references: (1) the combination of pulsed electrolysis and pulsed ultrasound [36, 37, 40]; (2) the combination of pulsed [34] or cyclic [39, 41] electrolysis and stationary ultrasound; and (3) synthesis at constant values of the electrode potential or current density and constant values of ultrasound parameters [35, 39]. Precursors of silver are mainly the soluble salts, such as AgNO_3_ [34, 36, 40], Ag_3_C_6_H_5_O_7_ [37], and AgClO_4_ [39]. The use of sacrificial silver anode is promising to ensure a stable concentration of Ag(I) ions and, accordingly, the efficacy of sonoelectrochemical synthesis of AgNPs [37, 41]. It was reported [41] that, in solutions of polymeric surfactant (polyacrylate), the currents of anodic dissolution of silver with the formation of complexes [(Ag^+^)_m_PА]^(n−m)^ (equation (8)) are commensurate with the cathodic currents of reduction reaction (equation (9)). Also, taking into account the reactions (1–5) caused by ultrasound, the algorithm “*anodic dissolution–reduction of Ag(I)*–*nucleation and formation of AgNPs*” is provided. This causes the low concentrations of [(Ag^+^)_m_PА]^(n−m)^ complex ions in solution, which creates favorable conditions for the formation of small-sized silver nanoparticles (Figure 7):

(8) $$\begin{array}{c} \text{mAg}+{\text{PA}}^{\text{n}-}⟶{\left[\left({\text{Ag}}^{+}\right)\text{mPA}\right]}^{\left(\text{n}-\text{m}\right)}+\text{me} \end{array}$$

(9) $$\begin{array}{c} {\left[\left({\text{Ag}}^{+}\right)\text{mPA}\right]}^{\left(\text{n}-\text{m}\right)-}+\text{me}⟶{\left[\left({\text{Ag}}^{0}\right)\text{mPA}\right]}^{\text{n}-} \end{array}$$

#### 2.1.3. AuNPs

Sonoelectrochemical synthesis of AuNPs is carried out mainly in solutions containing the surfactants [43, 46–49] and in some cases without them [44, 45]. AuNPs synthesized without surfactants may be used in biomedicine and catalysis. Sacrificial gold anodes also are used [45–49].

A study of sonoelectrochemical synthesis of AuNPs without a stabilizer [44] demonstrated that the current density in a wide range of values has little effect on the UV-Vis spectra of colloid solutions and the geometry of nanoparticles. However, the effect of the current pulse duration is significant, with the increase in which there is a tendency to increase the size of nanoparticles (Figure 8).

In another study [47], a method of sonoelectrochemical synthesis of AuNPs by the dissolution of Au substrates via electrochemical treatments of “oxidation–reduction” cycles with subsequent sonoelectrochemical reductions of Au-ions to synthesize Ch/Au nanocomposite was proposed. Such Ch/Au nanocomposite can be destroyed in the ultrasonic field, and AuNPs are formed. Therefore, chitosan was included as a polymeric surfactant performing the function of a matrix during synthesis. The overall process can be represented by the algorithm: “*gold*_*polycrystalline*_* + Cl*^*−*^* + Ch*^*ORC*^* ⟶ Ch−[AuCl*_*4*_*]*^*−*^^*sonoelectrochem*^* ⟶ Ch−AuNPs*^*sonification*^* ⟶ AuNPs*,” which makes it possible to obtain the nanoparticles with the size of ∼12 nm and narrow size distribution. So, ultrasound performs a dual function in the proposed method of synthesis: the first is the promotion of the AuNPs formation during the electrochemical reduction of Ch−[AuCl_4_]^−^ and the second is the destruction of the formed Ch−AuNPs nanocomposites.

#### 2.1.4. PdNPs and PtNPs

In [50], it was shown that controlled sonoelectrochemical synthesis of PdNPs is affected by the following parameters, namely, current density, power of ultrasound, and surfactant concentration. It was shown that, with increasing the current density, the size of nanoparticles is decreased. Specifically, at і_cathode_ equal to 8 and 13 mА·сm^−2^, the diameters of formed PdNPs were equal to 10 and 5 nm, respectively. The optimal range of ultrasound power also has been determined. Under intensities lower than 20 W·cm^−2^, the particles were irregularly shaped and ere agglomerated due to insufficient ultrasound energy for effective ablation of PdNPs from the cathode surface. Hence, some of them continued to grow in the next cycle of cathodic reduction. The power range from 20 to 80 W·cm^−2^ was effective for obtaining PdNPs with a diameter from 5 to 10 nm. Using the intensities above 120 W·cm^−2^ was also problematic due to the local overheating of the cathode surface (up to 90°C), which causes the agglomeration of nanoparticles. Also, it has been shown that a surfactant should be present to prevent the agglomeration of nanoparticles. Another study [51] also revealed a similar trend to PdNPs size dependence on the value of current density.

A significant feature of sonoelectrochemical synthesis [52] is the formation of 3D dendritic structures of platinum with a diameter of about 30 nm. The authors showed the possibility of controlled influence of synthesis parameters on the size and morphology of nanoparticles. As specific example, it was reported that, at 5 mА·сm^−2^, monodispersed PtDPNs with size of 6 nm were formed; at 20 mА·сm^−2^, heterogeneous PtDPNs with broad variation in size were formed; and finally at 40 mА·сm^−2^, agglomeration of DPNs was observed. Another study [53] emphasized the importance of optimization of the duration of the electrochemical pulse for obtaining the desired size of PtPNs. It was shown that an increase in *τ*_on_ leads to an increase in the size of nanoparticles and also causes difficulties in PtPNs ablation from the surface of the sonoelectrode.

#### 2.1.5. FeNPs

In [54], the synthesis of FeNPs in tetrahydrofuran and atmosphere of argon was described, and the molecules of solvent [(C_4_H_9_)_4_N] play the role of the nanoparticles stabilizer. The size of FeNPs was regulated by the frequency of ultrasound during the electrochemical synthesis. It was found that, under the action of ultrasonic of 200 kHz and 20 kHz and simultaneous action of 200 and 20 kHz, the average sizes of the obtained iron particle were 29, 18, and 7 nm, respectively. The authors explain this as in the case of only low-frequency ultrasound at 20 kHz, an area of intense cavitation in the interelectrode space is formed. The cavitation effect is continued after the shaking of FeNPs from the surface of the sonocathode also in the volume of the solution, and this promotes the formation of smaller nanoparticles. At high frequencies (200 kHz), the cavitation effect occurs mainly on the cathode surface. Moreover, simultaneous use of low- and high-frequency ultrasonic fields can, in addition to cavitation, create both microflows of significant intensity and large-scale ultrasonic flows. This simultaneous action of low and high frequency ultrasonic fields increases the efficiency of the ultrasonic action in the liquid and leads to decreasing of the size of formed FeNPs.

In aqueous solutions, the sonoelectrochemical synthesis of FeNPs is based on the simultaneous cathodic reduction of Fe(+2) and H(+), where the formed H_2_ bubbles, in addition to providing a reducing atmosphere, affect the formation of nanoparticles [55].

#### 2.1.6. WNPs

Tungsten cannot be reduced in aqueous solutions, and hence the method of pulsed sonoelectrochemical coprecipitation of Fe and W can be used [57]. The process occurs due to the catalysis of reduction of tungsten (equation (11)) by the formed iron (equation (10)) with the formation of nanoparticles of FeWNPs. After ultrasonic ablation of particles from the cathode surface, FeWNPs in acidic solution are converted into WNPs due to the dissolution of iron:

(10) $$\begin{array}{c} {\left[{\text{FeC}}_{6}{\text{H}}_{5}{\text{O}}_{7}\right]}^{-}+2\text{e}⟶\text{Fe}+{\text{C}}_{6}{\text{H}}_{5}{\text{O}}_{7}^{3-} \end{array}$$

(11) $$\begin{array}{c} {\left[{\text{WO}}_{2}{\text{C}}_{6}{\text{H}}_{5}{\text{O}}_{7}\right]}^{-}+4{\text{H}}^{+}+6\text{e}⟶\text{W}+{\text{C}}_{6}{\text{H}}_{5}{\text{O}}_{7}^{3-}+2{\text{H}}_{2}\text{O} \end{array}$$

#### 2.1.7. MgNPs and AlNPs

Magnesium and aluminum are metals that can be reduced only in a nonaqueous medium due to their standard electrode potentials being equal to −2.356 V and −1.66 V, respectively. Therefore, the synthesis of MgNPs [58] and AlNPs [59] can be performed by the sonoelectrochemical method in an organic aprotic solvent (THF), which, in addition to the nonaqueous medium, acts as a stabilizer. Due to the donor-acceptor binding (CH_2_)_4_O: *⟶* Mg(Al), molecules of THF form surface complexes. This provides “encapsulation” of MNPs, preventing their agglomeration. The main function of the pulsating ultrasound was to shake the metal nanoparticles deposited on the cathode. Taking into account the requirement in MgNPs and AlNPs in the production of hydride materials based on these metals, the proposed techniques are considered suitable for use on a technological scale [58, 59].

### 2.2. Sonoelectrochemical Synthesis of M1M2NPs

In the case of composites, the coreduction of M_1_ and M_2_ is performed from solutions containing ions of two corresponding metals (Table 2). For metals which are a little differed in the values of standard electrode potentials (Fe, Co, Ni), the controlled content of components in M_1_M_2_NPs can be decided by controlling the concentrations of salts [56, 60–62]. Thus, sonoelectrochemical synthesis from FeSO_4_ + CoSO_4_ solutions of different concentrations makes it possible to obtain Fe_75_Co_25_NPs [60], Co_65_Fe_35_ [61], FeCo_(1–2)_NPs [62], and FeCo_(1–4)_NPs [62]. In the case of metals with large differences in the values of Δ*E*^0^ (Cu and Ni [64], Cu and Pt [65], Pd and Fe [66]), an advanced reduction of more electrodegradable metal is observed. For example, during the sonoelectrochemical synthesis of Cu-Pt nanopowders [65], part of the reduced copper acts as a sacrificial metal to reduce platinum (equation (12)). This allows synthesizing the Cu@PtNPs. In addition (equation (12)), the process of leaching copper from Cu-Pt nanopowders by reaction (13) is used to increase the platinum content. The combination of concentrations of precursors and processes (equations (12) and (13)) allows controlling the composition of particles: Cu_55_Pt_45_, Cu_25_Pt_75_, and Cu_42_Pt_58_:

(12) $$\begin{array}{c} \text{Pt}\left(\text{IV}\right)+2\text{Cu}⟶2\text{Cu}\left(\text{II}\right)+\text{Pt} \end{array}$$

(13) $$\begin{array}{c} \text{Cu}+\frac{1}{2}{\text{O}}_{2}+2{\text{H}}^{+}⟶{\text{Cu}}^{2+}+{\text{H}}_{2}\text{O} \end{array}$$

Similarly, WCoNPs can be obtained using the electrochemical reduction of tungsten from the tungstate ion WO_4_^2−^, which occurs due to catalysis by the citrate complex [Co(II)(C_6_H_5_O_7_)WO_2_]^−^_(ads)_ formed during the sonoelectrolysis [68].

In the sonoelectrochemical syntheses of M_1_M_2_NPs described in [60, 61, 63, 65–68], preferably the sizes of several nanometers are obtained. This is facilitated by the factor of alternate reduction of metals M_1_ and M_2_, that is, the deposition of each of them on a foreign surface. The synthesis is carried out mainly in solutions without surfactants (Table 2), and hence the products are obtained as agglomerates of M_1_M_2_NPs [56, 60–67].

## 3. Synthesis of Metallic Nanoparticles by Galvanic Replacement in Ultrasound Field

The process of galvanic replacement (according to the generalized equation (14)) takes place via the electrochemical mechanism [69–72], where ionization of the sacrificial metal M_1_ with “generation” of electrons (15) takes place at the anode areas and the reduction of M_2_^n+^ ions (16) occurs at the cathode sites:

(14) $$\begin{array}{c} {\text{mM}}_{2}^{\text{n}+}+{\text{nM}}_{1}⟶{\text{nM}}_{2}+{\text{nM}}_{1}^{\text{m}+} \end{array}$$

(15) $$\begin{array}{c} \text{anode}:{\text{M}}_{1}⟶{\text{M}}_{1}^{\text{m}+}+{\text{me}}^{-} \end{array}$$

(16) $$\begin{array}{c} \text{cathode}:{\text{M}}_{2}^{n+}+{\text{ne}}^{-}⟶{\text{M}}_{2} \end{array}$$

Depending on the nature of the sacrificial metal pair “*sacrificial (M*_*1*_*) – reduced (M*_*2*_),” the formation of sediments of the following three types is possible: the islands, the dendritic, and the film. The first two types are of the greatest interest for obtaining metal nanoparticles. The formation of “island” sediment occurs with a significant difference between the crystal lattices M_1_ and M_2_ and is realized according to the Volmer–Veber mechanism [75]. For example, the galvanic replacement of metals on the surfaces of magnesium [72] and silicon [71, 73] can be considered. The formation of dendritic sediment occurs at a high rate of the process (equation (14)), which is primarily due to the significant difference between the values of standard electrode potentials between M_1_ and M_2_ [72–75]. However, galvanic replacement is mainly used to extract metals from leaching solutions of ore and secondary raw materials. In the last decade, the galvanic replacement method has been intensively studied as effective for surface modification by metal nanoparticles and nanostructures [69–73].

The use of ultrasound significantly accelerates the rate of galvanic replacement, primarily due to the acceleration of the electron-generating reaction (equation (15)) because of the intensive renewal of the anode areas and the prevention of their passivation. Therefore, at the corresponding ultrasound parameters, as well as in solutions containing the surfactants, MNPs and M_1_M_2_NPs are obtained via the galvanic replacement technique (Table 3). In addition, ultrasound, by analogy with sonoelectrochemical syntheses, performs the function of “shaking” of MNPs from the cathode regions of the sacrificial metal. Surfactants, due to adsorption and formation of surface complexes with MNPs, inhibit their growth during the galvanic replacement and prevent the agglomeration of particles in solutions (Figure 9). Therefore, it is possible to obtain the MNPs with a small mean size (up to 10 nm) and narrow size distribution. Specifically, the example of galvanic replacement of gold and platinum [78] showed that acoustic cavitation causes rapid nucleation, which contributes to the formation of a large number of MNPs with a uniform size distribution over a short period of time (usually several minutes). Simultaneously with ultrasound galvanic substitution, the formation of MNPs can also occur using the sonochemical reactions (4–6), since cavitation induces the formation of H· and HO· and other secondary radicals that reduce metal ions in solutions. However, such parallel processes are not described in the literature. Using ultrasound galvanic replacement, stabilized MNPs were synthesized (M = Fe, Co, Sn, Cu, Ag, Au, Ru, Pt) in PVP solutions [76, 78, 79]. Compact metal samples, among which the active ones such as magnesium, aluminum [79], as well as iron [78], copper [76, 78], and silver [77], were used as sacrificial templates for the synthesis of nanoparticles.

In the literature, the ultrasound galvanic replacement techniques have been demonstrated for obtaining of core@shell nanoparticles M_1_@М_2_NPs [82, 84, 86] and nanoalloys M_1_М_2_NPs [80, 81, 83, 85]. In [86], a hybrid method of Pd@Pt core-shell nanoparticles synthesis was proposed. In accordance with this method, the ultrasound is used for the realization of two successive processes: first is the sonochemical synthesis of PdNPs in PdCl2 solutions followed by the second one which is the galvanic substitution of platinum on the surface of palladium nanoparticles (Figure 10).

## 4. Conclusions

The combination of electrochemical reduction and ultrasonic field in aqueous solutions allows carrying out the controlled synthesis of metal nanoparticles with given geometry and bimetallic nanoparticles with controlled composition. Sonoelectrochemical synthesis, as a hybrid technique, is characterized by a high rate of nucleation and formation of MNPs and M_1_M_2_NPs with the minimum number of precursors and controllability. Therefore, it can be attributed to the “green” and promising technologies of nanomaterials production. The use of sacrificial anodes provides an algorithm “*anodic dissolution–electrochemical reducing of metal−nucleation and growth of МNPs*” which allows the design of nanoparticles.

Galvanic replacement under ultrasonic field in solutions containing the surfactants allows synthesizing stabilized MNPs. Sonogalvanic replacement is an effective method for obtaining nanoalloys (M_1_M_2_NPs) and core@shell nanoparticles (M_1_@M_2_). The processes at the anode and cathode areas of sacrificial metals in ultrasound are similar to the processes occurring at the sonoelectrochemical synthesis of MNPs due to the electrochemical nature of galvanic replacement.

## Figures and Tables

**Figure 1:** Applications of silver nanoparticles in biomedicine reproduced from [2] under the terms of the creative commons CC BY license.

**Figure 2:** The unique attributes of AuNPs reproduced from [7] under the terms of the creative commons CC BY license.

**Figure 3:** TEM images of AgNPs synthesized in solution NaPA (5 g L-1) by cyclic voltammetric (during 20 cycles) without ultrasonic field (a) and in the ultrasonic field (b), *t* = 20°C. Reproduced from [41] under the terms of the Creative Commons CC BY license.

**Figure 4:** Scheme of pulsed current supply and ultrasound during sonoelectrochemical synthesis of MNPs.

**Figure 5:** Scheme of MNPs formation by pulsed current supply and pulsed ultrasound in solution with surfactant.

**Figure 6:** Scheme of formation of complexes of Ag(+) ions with PVP (a) or PA^−^ (b).

**Figure 7:** TEM images (a) and the size distribution histograms (b) of AgNPs, synthesized in RL solution (2 g/L) at 40 cycles, *t* = 20°C. Reproduced from [42] under the terms of the Creative Commons CC BY license.

**Figure 8:** TEM images of the Au NPs synthesized by sonoelectrochemical method at different pulse times (*τ*_current_/*τ*_sono_). (a) 0.3 s/0.3 s. (b) 0.4 s/0.4 s. (c) 0.5 s/0.5 s. (d) 1.0 s/1.0 s. Reproduced from [44] under the terms of the Creative Commons CC BY license.

**Figure 9:** Scheme of MNPs formation by galvanic replacement and ultrasound in solution with surfactant.

**Figure 10:** Schematic illustration for the synthesis of Pd@Pt core shell using ultrasonication. Reproduced from [86] under the terms of the Creative Commons CC BY license.

**Table 1:** Conditions of the sonoelectrochemical synthesis of metal nanoparticles (MNPs).

MNPs	Precursors	Surfactant	i_сathode_, mA·cm^−2^ or E	Ultrasonic frequency (kHz)	Ultrasonic power	*λ*_max_ (nm)	Particle size (nm)	Refs.

CuNPs	CuSO_4_ + H_2_SO_4_	PVP (10000)	50–200	20, *τ*(US)_on_ = 5 s *τ*(US)_off_ = 3 s	40 W	—	15–900	[30]
	CuSO_4_ + H_2_SO_4_	PVA (100000)	—	20, *τ*(US)_on_ = 0.25 s, *τ*(US)_off_ = 0.3 s	—	589, 616, 626	8.5 ± 1.5 in dendrite	[31]
	CuSO_4_ + H_2_SO_4_	PVP (8000–35000)	500–1000	22	—	—	∼100	[32]
	CuSO_4_ + H_2_SO_4_	PVP (4000)	480, *τ*_on_ = 0.25 s, *τ*_off_ = 0.25 s	20, *τ*(US)_on_ = 0.1 s, *τ*(US)_off_ = 0.15 s	—	589	25–60	[33]

AgNPs	AgNO_3_	NTA	50, *τ*_on_ = 0.3 s, *τ*_off_ = 0.6 s	—	60 W·cm^−2^	413	Nanorods, Φ = 10–20	[34]
	AgNO_3_	EDTA	40	50	100 W	—	Φ = 80, >15 *μ*m long	[35]
	AgNO_3_	NTA	50, *τ*_on_ = 0.6 s, *τ*_off_ = 0.6 s	*τ*(US)_on_ = 0.3 s, *τ*(US)_off_ = 0.9 s	750 W	—	5 ± 2, 60 ± 30, 75 ± 25	[36]
	Ag_3_C_6_H_5_O_7_ + NaAc^−^HAc	PVP (40000)	70, *τ*_on_ = 3 s, *τ*_off_ = 3 s	20, *τ*(US)_on_ = 3 s, *τ*(US)_off_ = 3 s		410	20–25	[37]
	Sacrificial silver anode in HCl	Without stabilizer	Ag electrode was cycled in 0.1 M HCl −0.3…+0.3 V	20	100 W	410	2–20	[38]
	AgClO_4_	PVP (49000)	CV, 0.25–2.00	40	50 W	415–426	7–10	[39]
	AgNO_3_	SDS	20, *τ*_on_ = 0.3 s, *τ*_off_ = 0.9 s	*τ*(US)_on_ = 0.3 s, *τ*(US)_off_ = 0.6 s	100 W·cm^−2^	401, 418	∼20	[40]
	Sacrificial silver anode	NaPA	CV 50 mV·s^−1^, E from 1.0 to −1.0 V	22	40–62.5 W·dm^−3^	500	4–30	[41]
	Sacrificial silver anode	Rhamnolipid	CV 50 mV·s^−1^, E from +1.0 to −1.0 V	22	40–62.5 W·dm^−3^	415	1–3	[42]

AuNPs	H[AuCl_4_]	MPEO/PVP	−850 …−1300 mV;*τ*_on_ = 10–20 ms, *τ*_off_ = 200–300 ms	27	—	520; 550	5–35	[43]
	H[AuCl_4_] + KNO_3_	Without stabilizer	16,3	20, *τ*(US)_on_ = *τ*(US)_off_ = 0.5 s	20 W	500–556	10–100	[44]
	Sacrificial gold anode in HCl	Without stabilizer	0.2, 0.4, and 0.6 V	20	100 W		2–15	[45]
	Sacrificial gold anode	Ch	ORC, from −0.28 to +1.22 V	20	100 W	520–533	5 ± 2	[46]
						522, 531	12	[47]
						522, 530	15	[48]
		CTAB	ORC, from −0.28 to +1.22 V	20	100 W	518, 521	5	[49]

PdNPs	PdCl_2_	CTAB	8…13, *τ*_on_ = *τ*_off_ = 5…10 s	20	20–80, 120 W·cm^−2^	—	5–13	[50]
	H_2_[PdCl_4_] + KNO_3_	CTAB, PVP	25, *τ*_on_ = *τ*_off_ = 0.5 s	20, *τ*(US)_on_ = 0.3 s, *τ*(US)_off_ = 0.7 s	20 W	—	7	[51]

PtDPNs	H_2_[PtCl_6_] + KNO_3_	PVP (40000), SDS	10, *τ*_on_ = 1.0 s, *τ*_off_ = 0.5 s	20, *τ*(US)_on_ = 0.3 s, *τ*(US)_off_ = 1.5 s	20 W	—	Nanodendrites with primary NPs 2.5 ± 0.5	[52]

PtNPs	K_2_[PtCl_4_] + NaCl	—	50, *τ*_on_ = 0.3 s, *τ*_off_ = 0.6 s	20, *τ*(US)_on_ = 0.3 s, *τ*(US)_off_ = 0.6 s	70 W	—	11–15	[53]
FeNPs	Sacrificial iron anode	THF, (C_4_H_9_)_4_NBr	16	200 on cathode; 20 kHz on horn	1.5 W·cm^−2^ cathode; 50 W·cm^−2^ horn	—	∼29, ∼18, ∼7	[54]
	FeCl_2_	—	4–240	4	—	—	Nanodendrites with crystallites 10–100	[55]

NiNPs	NiSO_4_ + NH_4_Cl + H_3_BO_3_ + C_6_H_8_O_7_	—	2000 A·m^−2^ *τ*_on_ = 1–1000 ms, *τ*_off_ = 100–1000 ms	20, *τ*(US)_on_ = 100–1000 ms	50 W·cm^−2^	—	50	[56]
WNPs	Na_2_WO_4_ + FeSO_4_ + Na_3_C_6_H_5_O_7_ + C_6_H_8_O_7_	—	7·10^4^ A·m^−2^	10 Hz and the dead time of 0.09 s	500 kW·m^−2^	—	∼30	[57]
MgNPs	RMgCl + AlCl_3_ in THF	THF, DBDG	—	—	—	—	4.5 ± 0.5	[58]
AlNPs	AlCl_3_ + LiAlH_4_ in THF	THF	100 mAcm^−2^, *τ*_on_ = 600 s, *τ*_off_ = 60 s	20, *τ*(US)_on_ = 240 ms	76 W	—	10–20	[59]

**Table 2:** Conditions of the sonoelectrochemical synthesis of bimetal nanoparticles (M_1_M_2_NPs).

M_1_M_2_NPs	Precursors	Surfactant	i or E	Ultrasonic frequency (kHz)	Ultrasonic power	Particle size (nm)	Refs.

(CoNi)NPs (FeNi)NPs (FeCo)NPs	(Co, Ni, Fe)SO_4_ + NH_4_Cl + H_3_BO_3_	—	8000 A·m^−2^, *τ*_on_ = *τ*_off_ = 300 ms	20, *τ*(US)_on_ = 200 ms	50 W·cm^−2^	∼100	[56]
Fe_75_Co_25_	FeSO_4_ + CoSO_4_ + NH_4_Cl + H_3_BO_3_ + C_6_H_8_O_7_	—	−3.0…−4.5 V	20	50 W·cm^−2^	2–4 in agglomerate 30 nm	[60]
Co_65_Fe_35_	FeSO_4_ + CoSO_4_ + NH_4_Cl + H_3_BO_3_ + C_6_H_8_O_7_	—	*τ*_on_ = 0.3 s, *τ*_off_ = 0.5 s	20, *τ*(US)_on_ = 0.5 s, *τ*(US)_off_ = 0.3 s	118 W·cm^−2^	NPs ∼5 nm in clusters ∼300 nm	[61]
FeCo	FeSO_4_ + CoSO_4_ + NaCl + H_3_BO_3_	Without stabilization and stabilization by NaPA	80 mA·cm^−2^ *τ*_on_ = 0.35 s, *τ*_off_ = 0.75 s	20, *τ*(US)_on_ = 0.3 s, *τ*(US)_off_ = 0.7 s	76 W	8.6 ± 0.3 (10°C), 12.3 ± 0.5 (25°C), 25.1 ± 1.3 (40°C), 28.1 ± 1.4 (60°C)	[62]
FeCr	FeCl_2_ + CrCl_3_ + NH_4_Cl + H_3_BO_3_ + glycine	—	120 mA·cm^−2^	20	75 W·cm^−2^	4,6 ± 0,2 (25°C), 5 ± 0,1 (40°C)	[63]
CuNi	NiSO_4_ + CuSO_4_ + Na_3_C_6_H_5_O_7_	—	100 mA·cm^−2^, *τ*_on_ = 0.3 s, *τ*_off_ = 0.7 s	20, *τ*(US)_on_ = 0.3 s, *τ*(US)_off_ = 0.5 s	75 W	∼15	[64]
CuPt	CuSO_4_ + H_2_SO_4_ + Na_2_[PtCl_6_]	—	*E* = −1.0 V, *τ*_on_ = 100 ms, *τ*_off_ = 200 ms	24, *τ*(US)_on_ = 100 ms, *τ*(US)_off_ = 200 ms	100 W·cm^−2^	9 ± 4 for Cu_42_Pt_58_. ∼10 for Cu_65_Pt_35_	[65]
PdFe	FeSO_4_ + PdCl_2_ + H_3_BO_3_	—	2500–5500 A·m^−2^, *τ*_on_ = 100 ms, *τ*_off_ = 200 ms	20	50 W·cm^−2^	Agglomerates 50–100 nm, with individual NPs ∼5 nm	[66]
AuAg	[AuCl_4_]^−^ + [AgCl_2_]^−^	—	*E* = −0.75 V	20	100 W	∼5	[67]
WCo	CoSO_4_ + Na_2_WO_4_ + Na_3_C_6_H_5_O_7_	SDS	*τ*_on_ = 500 ms, *τ*_off_ = 800 ms	38	80 W	100–500 ratio of W : Co in NPs was 23 : 4	[68]

**Table 3:** Conditions of the synthesis of metallic nanoparticles (MNPs, М_1_М_2_NPs) by galvanic replacement in an ultrasonic field.

Metallic nanoparticles	Sacrificial metal	Surfactant	Precursor of MNPs	Ultrasonic parameters	*t*, °C	Time of GR	Size of NPs (nm)	Refs.

*MNPs*								
AgNPs, Ag nanodendrites	Cu sheet	PVP	AgNO_3_	40 kHz	22 ± 2	10 min	100	[76]
Nano-/microporous Au microsheets	Ag plate	—	H[AuCl_4_]	135 W	22 ± 2	10 min	30–60	[77]
AuNPs	Cu foil	PVP	H[AuCl_4_]	42 kHz		5 min	10	[78]
PtNPs	Fe foil	PVP	H_2_[PtCl_6_]	42 kHz		10 min	10	[78]
RuNPs (Ag, Cu, Fe, Co, Ru, and Sn)	Mg foil (Al, Co)	PVP	RuCl_3_	42 kHz 70 W		4 min	3.1 ± 0.9	[79]

*M*_*1*_ *M*_*2*_ *NPs*								
CuAgNPs	СuNPs		Ag_2_O	80 W	30	5 min	10–80	[80]
CuAgNPs	СuNPs		Ag_2_O	100 W/сm^−2^	22 ± 2	—	5–10	[81]
Pd@CuNWs/MWCNTs-CH	Cu NWs		PdCl_2_		22 ± 2	1 hour	150	[82]
Pd-AgNPs	Ag		PdCl_2_	40 MHz	25	5 min	2–3	[83]
Ni@PtNPs	NiNPs		Pt(acac)_2_	20 kHz	22 ± 2	3 hr	3–4	[84]
PtCuNPs/NCNT	CuNPs/NCNT	—	Pt(NO_3_)_2_	100 W, 20 kHz	22 ± 2	3 min	≤5	[85]
Pd@Pt/CNPs	Pd	SDS	H_2_[PtCl_6_]	20 kHz	25 ± 1	20 min	3–5	[86]

## Abbreviations

Ch: Chitosan
CTAB: Cetyltrimethylammonium bromide
DBDG: Dibutyl diglyme
DPNs: Dendritic particles nanostructures
*E* ^0^: Standard electrode potential
i_сathode_: Cathode current density
MNCs: Metal nanoclusters
MNPs: Metal nanoparticles
MPEO-SH: M a-Methoxy-x-mercapto-poly(ethylene oxide)
NaPA: Sodium polyacrylate
NTA: N(CH_2_COOH)_3_, nitrilotriacetate
ORC: Oxidation-reduction cycles
PDDA: Polydiallyldimethylammonium chloride
PVA: Polyvinyl alcohol
PVP: Polyvinylpyrrolidone
SDS: Sodium dodecyl sulfate CH_3_(CH_2_)_11_OSO_3_Na
THF: Tetrahydrofuran
US: Ultrasound.
